# Occupational Stress and Insomnia Symptoms Among Nurses During the Outbreak of COVID-19 in China: The Chain Mediating Effect of Perceived Organizational Support and Psychological Capital

This article has been retracted.

**DOI:** 10.3389/fpsyt.2022.882385

**Published:** 2022-07-07

**Authors:** Juan Du, Zhuo Liu, Xuejing Zhang, Pei Shao, Yan Hua, Yang Li, Hongjuan Lang, Chunping Ni

**Affiliations:** ^1^School of Nursing, The Fourth Military Medical University, Xi'an, China; ^2^School of Nursing and Rehabilitation, Shandong University, Jinan, China

**Keywords:** effort reward imbalance, overcommitment, perceived organizational support, psychological capital, occupational stress, insomnia symptoms

## Abstract

**Background:**

Nurses play an important role in medical and health services and insomnia symptoms were relatively high among nurses, especially during the epidemic of 2019 coronavirus disease. Insomnia not only damages the physical and mental health of the individual, but also reduces the efficiency of their work and the quality of care, ultimately impacting on patient care.

**Objective:**

The purpose of this study was to explore the role of perceived organizational support and psychological capital in the relationship between occupational stress and insomnia among Chinese nurses.

**Methods:**

A cross-sectional study has been carried out in a tertiary grade A hospital in Shandong Province, China from March 2021 to May 2021. The self-administered questionnaires were distributed to 810 nurses, which including Chinese Effort-Reward Imbalance Scale, Athens Insomnia Scale, Perceived Organizational Support Questionnaire, Chinese Psychological Capital Questionnaire, gender, age, education level and other demographic characteristics. Effective respondents were 658 (81.2%). Descriptive analysis, independent-samples *t*-test, one-way analysis of variance, Pearson correlation analyses, ordinary least-squares regression and the bootstrap method were used for data analysis.

**Results:**

The prevalence of insomnia symptoms in this study was found to be 57.3%. There were significant differences in insomnia symptoms in weekly working hours (*t* = −2.027, *P* = 0.043), with chronic disease (*t* = −2.825, *P* = 0.005), negative life events (*t* = −5.340, *P* < 0.001), departments (*F* = 3.077, *P* = 0.006) and position (*t* = 2.322, *P* = 0.021) among nurses. Overall, the serial-multiple mediations of perceived organizational support and psychological capital in the relationship between occupational stress and insomnia were found to be statistically significant.

**Conclusions:**

The prevalence of insomnia symptoms was comparatively high among Chinese nurses, and occupational stress had direct negative influence on it. Perceived organizational support and psychological capital acted as chained mediating factor could partially relieve insomnia symptoms related to occupational stress. Supportive working environment should be provided, and improving psychological capital levels to help nurses coping with insomnia symptoms.

## Introduction

The epidemic of 2019 coronavirus disease (COVID-19) has exacerbated occupational stress of medical staff in the worldwide, resulting in psychological distress and stress-related health behavior problems (1–5). Nurses who are predominantly female are more likely to have mental problems. They still need to undertake most public health tasks such as nucleic acid testing in high and medium-risk areas to improve case identification and vaccination when the epidemic is stabilizing in China. Insomnia is one of the psychological problems. Several studies have shown that insomnia symptoms were observed in 34.0–40.1% of health care workers during the COVID-19, with nurses having the highest prevalence (2, 6–8). The global nursing workforce shortage (9), increasing demand for care, long-term high workload, high risk, irregular work rhythm and tense nurse-patient relationship may lead to potential occupational stress, which is the main cause of insomnia among nurses. Insomnia leads to impaired attention, decision-making ability and thinking flexibility of nurses, which has a significant impact on nurses' work performance and poses a threat to patients' safety (10).

It has been reported that occupational stress was significantly associated with insomnia (11–13). A cross-sectional study involving 3,013 nurses in Brazil found that occupational stress increased the odds of insomnia by 2.2 times (14). Effort-Reward Imbalance (ERI) Model was widely used to study the relationship between job characteristics and employee health. From the perspective of social exchange theory, the ERI model explores the mechanism of occupational stress from three aspects of effort, reward and overcommitment. Studies have found that the occupational stress defined by ERI may be related to sleep disturbances through the cortisol elevation and the hypothalamic-pituitary-adrenal (HPA) axis activation (15, 16).

Positive factors existing in work environment, such as organizational support, played an important role in alleviating the occupational stress of employees and improving their mental health problems (4, 17). According to the job demands-resources (JD-R) model, the characteristics of any job can be divided into job demands and job resources (18). Job demands are factors that consume individual energy in work, such as work overload, role conflict and time pressure, etc. While organizational support is one of the positive factors that belong to work resources and can effectively reduce job demands and related psychological and physiological costs. Research by Zou et al. found that with increased organizational support, the risk of insomnia among frontline healthcare workers fighting against COVID-19 declined (19). Both the ERI and JD-R model suggest that occupational stress and lack of organizational support are important predictors of negative outcomes for individuals and organizations.

Xanthopoulou (20) incorporates psychological capital into the JD-R model, which was defined as the positive self-evaluation related to mental resilience and the psychological belief that one's own ability can successfully control and influence the environment. It mainly includes self-efficacy, hope, resilience, and optimism, has significant positive impact on employee's performance and satisfaction. Previous studies have found that both perceived organizational support and occupational stress affect psychological capital level of medical personal, and perceived organizational support was positively associated with psychological capital (21, 22).

Based on the theoretical perspectives and research conclusions presented above, exploring the modifiable work-related factors was essential to prevent and alleviate insomnia in nurses. The purpose of this study was to explore the role of perceived organizational support and psychological capital in the relationships between occupational stress and insomnia among Chinese nurses. There are four hypotheses proposed: (1) Occupational stress is positively correlated with insomnia. (2) Perceived organizational support plays a mediating role in occupational stress and insomnia. (3) Psychological capital plays a mediating role between occupational stress and insomnia. (4) Perceived organizational support and psychological capital play a chain mediating role between occupational stress and insomnia.

## Materials and Methods

The present study was approved by the Ethics Committee of the First Affiliated Hospital of Shandong First Medical University and complied with the Declaration of Helsinki. The purpose of this study was explained to all participants before conducting the survey and informed consent was also obtained.

### Study Design and Participants

This cross-sectional survey was conducted in Jinan city, Shandong Province, China, from March to May 2021. Cluster sampling procedures were used to recruit participants from a tertiary grade A hospital and a total of 810 nurses were recruited for the present study, 658 valid questionnaires were collected with an effective response rate was 81.2%. Inclusion criteria: (1) clinical registered nurse, and clinical nursing work for more than 1 year; (2) nurses gave informed consent and volunteer to participate in this study. Exclusion criteria: (1) nurses on sick leave or maternity leave during the study period; (2) advanced students or on-the-job logistics personnel. Once Institutional Review Board approval was obtained, anonymous questionnaires were sent out to nurses who met the inclusion and exclusion criteria by uniformly trained investigators, and standardized explanations were made if necessary.

### Measures

#### Basic Information

The self-developed demographic questionnaire included gender, age, education background, monthly income, working hours per week, chronic disease (“Do you have a chronic disease? If yes, what is it”), negative life events (“Have you experienced any of the following negative life events in the past year: health deterioration, financial difficulties, death of a loved one, loss of possessions, sad events, family conflicts, had difficulties with workmates, etc.”), department, and position (nurse or nurse manager).

#### Occupational Stress

The 23-item ERI scale was applied in this study (23), measuring extrinsic effort, reward and overcommitment. It uses a 5-point Likert scale, in which 1 indicates no stressful experience and 5 indicates the highest level of stressful experience. According to a predefined algorithm, Effort-Reward ratio (ERR) was calculated to quantify the degree of mismatch between high cost and low gain. Occupational stress can be expressed by ERR and overcommitment independently. The Chinese version of the ERI scale has been widely applied among Chinese occupational groups and found to have good reliability and validity (24). In this study, the Cronbach's alphas coefficient for the extrinsic effort, reward and overcommitment were 0.874, 0.941, and 0.915, respectively.

#### Measurement of Insomnia

Insomnia of nurses was measured by the Athens Insomnia Scale (AIS) (25). The AIS consists of eight items and each item was rated 0, 1, 2, and 3 from none to severe, and the range for insomnia is 0–24, with higher scores indicating poorer sleep quality. Participants were asked to choose a rating item only if they had experienced difficulty sleeping at least three times a week in the previous month. A total score of <4 was classified as no sleep disorder, and a score of 4–6 was classified as suspected insomnia, and a total score of more than 6 was classified as insomnia. The Chinese version of AIS has been found to have good validation (26). The Cronbach's alpha coefficient was 0.883 in this study.

#### Measurement of Perceived Organizational Support

Perceived Organizational Support Questionnaire was developed by Eisenberger et al. (27). A simplified Chinese version of the Perceived Organizational Support Questionnaire was applied and validated among Chinese occupational groups (28, 29). The questionnaire consists of 9 items, all items were scored on a 7-point Likert scale in which 1 representing completely disagreement and 7 representing completely agreement. Higher score indicates the stronger perceived organizational support. The Cronbach's alpha coefficient of the questionnaire in this study was 0.889.

#### Measurement of Psychological Capital

Psychological capital of nurses was measured by Psychological Capital Questionnaire (PCQ-24) (30). There were four dimensions with 6 items, respectively, including self-efficacy, hope, resilience and optimism, with each item was scored on a 5-point Likert scale, from 1 (strongly disagree) to 5 (strongly agree). Higher values indicated higher level of psychological capital. Studies have shown that the Psychological Capital Questionnaire has good reliability and validity under the cultural background of China (24). The Cronbach's alpha coefficient for the four dimensions of this questionnaire was 0.913, 0.907, 0.901, and 0.813, respectively. Cronbach's alpha coefficient for the PCQ-24 was 0.956 in this study.

### Statistics

Kolmogorov-Smirnov (K-S) single sample test and P-P diagram were used to test the Gaussian distribution of the data. Descriptive analysis was presented as counts (n) and percentages (%); independent-sample *t*-test and one-way analysis of variance (ANOVA) were used to compare the demographic data. Pearson correlation analyses of the four variables (occupational stress, perceived organizational support, psychological capital and insomnia) were performed. Model 6 in PROCESS macro developed by Hayes (31) was used to test the mediating effect of perceived organizational support and psychological capital in the relationship between occupational stress and insomnia, in which all statistically significant confounding factors in demographic analysis were taken as covariates in the analysis. This approach was based on ordinary least-squares regression and the bootstrap method. Hayes recommended 10,000 bootstrap bias-corrected 95% confidence intervals (BC CI) to be used for mediation analyses in the test from the Serial-Multiple Mediation Model 6, and if they did not contain zero, they were considered significant (31). The unstandardized path coefficients were calculated to reduce type 1 errors due to distribution. PROCESS macro was performed using one independent variable (ERR/overcommitment), two mediators (perceived organizational support and psychological capital), and one dependent variable (insomnia symptoms). SPSS 25.0 software was used for statistical analysis and the significance test level was *P* < 0.05.

## Results

In this study, of 810 selected subjects, 756 returned the questionnaire (response rate was 93.3%). After some subjects with missing values were excluded, the data from 658 subjects (81.2% of 810) were analyzed in this study.

### Preliminary Analyses

The demographic data and the distribution of insomnia symptoms are shown in Table 1. Data from 658 nurses were collected and the percentage of female in the study population was 83.4%; 71.9% were <30 years old; 78.0% had bachelor's degree; 51.5% earned between 5,000 and 8,000 RMB per month; 36.3% worked more than 40 h per week; 19.8% suffered from chronic diseases, 30.9% experienced negative life events, 32.4% were from surgery department, and 96.2% occupational position was nurse.

**Table 1:** Demographic statistics and the influence of demographic information and life behavior factors on insomnia.

**Variables**	**Number (*N*)**	**Percentage (%)**	**Insomnia**		***T*/*F***	***P***
			**Mean**	**SD**		
Gender					−0.001	0.999
Male	109	16.6	7.700	5.051		
Female	549	83.4	7.700	4.535		
Age (years)					0.371	0.690
<30	473	71.9	7.620	4.419		
30–40	132	20.0	8.010	5.379		
>40	53	8.1	7.620	4.395		
Education					1.413	0.244
Junior college and below	121	18.4	7.480	4.048		
College	513	78.0	7.810	4.705		
Postgraduate	24	3.6	6.290	5.377		
Monthly income (RMB)					1.587	0.205
≤ 5,000	213	32.4	7.400	4.601		
5,000–8,000	339	51.5	7.670	4.614		
>8,000	106	16.1	8.380	4.655		
Weekly working hours (hours)					−2.027	0.043
≤ 40	419	63.7	7.420	4.385		
>40	239	36.3	8.180	4.979		
With chronic disease					−2.825	0.005
No	528	80.2	7.420	4.449		
Yes	130	19.8	8.810	5.129		
Negative life events					−5.340	<0.001
No	455	69.1	7.070	4.441		
Yes	203	30.9	9.110	4.713		
Departments					3.077	0.006
Internal medicine	109	16.6	7.720	4.380		
Surgery	213	32.4	7.800	4.667		
Gynecology and obstetrics	61	9.3	6.230	4.656		
Pediatrics	42	6.3	7.070	5.004		
Emergency	39	5.9	9.080	4.515		
Operating room	84	12.8	6.870	3.751		
ICU	110	16.7	8.670	4.959		
Position					2.322	0.021
Nurse	633	96.2	7.780	4.628		
Nurse manager	25	3.8	5.600	3.969		

The prevalence of insomnia symptoms among Chinese nurses in this study was found to be 57.3%. There were significant differences in insomnia symptoms related to weekly working hours (*t* = −2.027, *P* = 0.043), with chronic disease (*t* = −2.825, *P* = 0.005), negative life events (*t* = −5.340, *P* < 0.001), departments (*F* = 3.077, *P* = 0.006), and position (*t* = 2.322, *P* = 0.021) among nurses.

### Preliminary Correlation Analyses

The means, standard deviations, and the correlations between variables are shown in Table 2. Results showed that insomnia symptoms were positively related to ERR (*r* = 0.379, *P* < 0.001), overcommitment (*r* = 0.466, *P* < 0.001), and negatively related to perceived organization support (*r* = −0.358, *P* < 0.001), self-efficacy (*r* = −0.343, *P* < 0.001), hope (*r* = −0.366, *P* < 0.001), resilience (*r* = −0.300, *P* < 0.001), optimism (*r* = −0.414, *P* < 0.001) and total psychological capital (*r* = −0.402, *P* < 0.001).

**Table 2:** Correlation analysis of occupational stress, perceived organizational support, psychological capital and insomnia.

	**Organization**					**Psychological**
**Variables**	**support**	**Psychological capital**				**capital**	**Occupational stress**		**Insomnia**
		**Self-efficacy**	**Hope**	**Resilience**	**Optimism**		**ERR**	**Overcommitment**	
1. Organization support	1								
2. Self-efficacy	0.437^***^	1							
3. Hope	0.406^***^	0.809^***^	1						
4. Resilience	0.320^***^	0.749^***^	0.830^***^	1					
5. Optimism	0.448^***^	0.578^***^	0.645^***^	0.619^***^	1				
6. Psychological capital	0.455^***^	0.891^***^	0.933^***^	0.907^***^	0.798^***^	1			
7. ERR	−0.318^***^	−0.206^***^	−0.231^***^	−0.203^***^	−0.338^***^	−0.275^***^	1		
8. Overcommitment	−0.328^***^	−0.274^***^	−0.315^***^	−0.235^***^	−0.378^***^	−0.339^***^	0.586^***^	1	
9. Insomnia	−0.358^***^	−0.343^***^	−0.366^***^	−0.300^***^	−0.414^***^	−0.402^***^	0.379^***^	0.466^***^	1
Mean	45.43	25.67	24.97	25.61	25.34	101.59	0.76	16.26	7.70
Standard deviation	9.83	4.92	4.95	4.83	4.56	17.02	0.42	5.61	4.62

*** *P < 0.001. ERR means Effort—Reward ratio*.

### Mediation Analyses

To determine the mediating effect of perceived organizational support and psychological capital in the relationship between occupational stress and insomnia symptoms. The analysis results of ERR on insomnia symptoms mediated by perceived organizational support and psychological capital (ERR model) are present in Figure 1 and Table 3. The whole regression equation was statistically significant (*R*^2^ = 0.300, *F* = 21.185, *P* < 0.001). The mediation analysis of overcommitment on insomnia symptoms (overcommitment model) are present in Figure 2 and Table 4. The whole regression equation was also statistically significant (*R*^2^ = 0.341, *F* = 25.589, *P* < 0.001).

**Figure 1:** Serial-multiple mediation of perceived organizational support and psychological capital in the relationship between ERR and insomnia symptoms with non-standardized beta values and standard error. ***P < 0.001. ERR means Effort-Reward ratio.

**Table 3:** Comparison of indirect effects of ERR on insomnia symptoms mediated by perceived organizational support and psychological capital.

	**Product of coefficients**		**Bootstrapping 95% BC confidence interval (CI)**		**Proportion of indirect effect**
	**Point estimate**	**Boot SE**	**BootLL CI**	**BootUL CI**	
**Effect**
Total indirect effect of X on Y	1.043	0.274	0.600	1.678	29.31%
Indirect effect 1: X → M1 → Y	0.411	0.150	0.165	0.753	11.55%
Indirect effect 2: X → M2 → Y	0.359	0.158	0.108	0.737	10.09%
Indirect effect 3: X → M1 → M2 → Y	0.273	0.088	0.143	0.480	7.67%
**Contrasts**
Model 1 vs. Model 2	0.051	0.209	−0.389	0.436	
Model 1 vs. Model 3	0.138	0.160	−0.174	0.463	
Model 2 vs. Model 3	0.086	0.147	−0.184	0.401	

*N = 658. Number of bootstrap samples for bias corrected bootstrap confidence intervals: 10,000. Level of confidence for all confidence intervals: 95%. X, ERR; M1, perceived organizational support; M2, psychological capital; Y, insomnia symptoms. Model 1, ERR—perceived organizational support—insomnia symptoms; Model 2, ERR—psychological capital—insomnia; Model 3, ERR—perceived organizational support—psychological capital—insomnia symptoms. LL, lower level; UL, upper level; ERR, Effort—Reward Ratio*.

**Figure 2:** Serial-multiple mediation of perceived organizational support and psychological capital in the relationship between overcommitment and insomnia symptoms with non-standardized beta values and standard error. **P < 0.01, ***P < 0.001.

**Table 4:** Comparison of indirect effects of overcommitment on insomnia symptoms mediated by perceived organizational support and psychological capital.

	**Product of coefficients**		**Bootstrapping 95% BC confidence interval (CI)**		**Proportion of indirect effect**
	**Point estimate**	**Boot SE**	**BootLL CI**	**BootUL CI**	
**Effect**
Total indirect effect of X on Y	0.083	0.015	0.056	0.114	23.25%
Indirect effect 1: X → M1 → Y	0.030	0.010	0.013	0.051	8.40%
Indirect effect 2: X → M2 → Y	0.035	0.010	0.018	0.056	9.80%
Indirect effect 3: X → M1 → M2 → Y	0.017	0.005	0.009	0.028	4.76%
**Contrasts**
Model 1 vs. Model 2	−0.005	0.015	−0.036	0.025	
Model 1 vs. Model 3	0.013	0.011	−0.008	0.035	
Model 2 vs. Model 3	0.018	0.009	0.002	0.037	

*N = 658. Number of bootstrap samples for bias corrected bootstrap confidence intervals: 10,000. Level of confidence for all confidence intervals: 95%. X, overcommitment; M1, perceived organizational support; M2, psychological capital; Y, insomnia symptoms; Model 1, overcommitment—perceived organizational support—insomnia symptoms; Model 2, overcommitment—psychological capital—insomnia; Model 3, overcommitment—perceived organizational support—psychological capital—insomnia symptoms; LL, lower level; UL, upper level*.

Total effects of ERR (*c* = 3.559, SE = 0.392, *t* = 9.089, *P* < 0.001; *R*^2^ = 0.212, *F* = 15.807, *P* < 0.001) and overcommitment (*c* = 0.357, SE = 0.029, *t* = 12.367, *P* < 0.001; *R*^2^ = 0.281, *F* = 23.000, *P* < 0.001) on insomnia symptoms were found to be significant, respectively (Step 1). In addition, ERR (*B* = −6.291, SE = 0.861, *t* = −7.306, *P* < 0.001; *R*^2^ = 0.157, *F* = 10.961, *P* < 0.001) and overcommitment (*B* = −0.522, SE = 0.066, *t* = −7.909, *P* < 0.001; *R*^2^ = 0.168, *F* = 11.875, *P* < 0.001) respectively, had a negative direct effect on perceived organizational support. ERR (*B* = −5.570, SE = 1.466, *t* = −3.798, *P* < 0.001) and overcommitment (*B* = −0.667, SE = 0.112, *t* = −5.945, *P* < 0.001) had negative direct effects on psychological capital, respectively. The direct effect of perceived organizational support as the first mediating variable on the second mediating variable of psychological capital in ERR model (*B* = 0.673, SE = 0.064, *t* = 10.452, *P* < 0.001) and in overcommitment model (*B* = 0.628, SE = 0.064, *t* = 9.840, *P* < 0.001) was also found to be significant, respectively (Step 2). A review of the direct effects of mediating variables on insomnia symptoms showed that the effects of perceived organizational support (*B* = −0.065, SE = 0.018, *t* = −3.574, *P* < 0.001) and psychological capital (*B* = −0.065, SE = 0.010, *t* = −6.246, *P* < 0.001) in ERR model, also perceived organizational support (*B* = −0.058, SE = 0.018, *t* = −3.278, *P* = 0.001) and Psychological Capital (*B* = −0.053, SE = 0.010, *t* = −5.212, *P* < 0.001) in overcommitment model were significant, respectively (Step 3). When occupational stress and the two mediating variables were simultaneously entered into the model (Step 4), the direct effect of ERR (c' = 2.516, SE = 0.389, *t* = 6.467, *P* < 0.001) and overcommitment (c' = 0.274, SE = 0.030, *t* = 9.194, *P* < 0.001) on insomnia symptoms were also found to be significant separately. Overall, these results revealed that serial-multiple mediation had occurred.

When taking into account all variables (including covariates) in the tested model, as seen in Tables 3, 4, the path through single mediation of perceived organizational support in ERR model [point estimate = 0.411; 95% Boot CI (0.165, 0.753)] and in the overcommitment model [point estimate = 0.030; 95% Boot CI (0.013, 0.051)], the path through single mediation of psychological capital in ERR model [point estimate = 0.359; 95% Boot CI (0.108, 0.737)] and in the overcommitment model [point estimate = 0.035; 95% Boot CI (0.018, 0.056)], and the path through both mediators in ERR model [point estimate = 0.273; 95% Boot CI (0.143, 0.480)] and in the overcommitment model [point estimate = 0.017; 95% Boot CI (0.009, 0.028)] were all statistically significant. The total indirect effect was also statistically significant in ERR model [point estimate = 1.043; 95% Boot CI (0.600, 1.678)] and in the overcommitment model [point estimate = 0.083; 95% Boot CI (0.056, 0.114)]. Thus, the path through both mediators was significant, moreover the indirect effect through both perceived organizational support alone and psychological capital alone was also significant.

In the present study, to decide whether specific indirect effects of mediators were stronger than others, contrasting findings were indicated, and three pairs of contrasting findings were found. In addition, as shown in Table 3, the three statistically significant contrasts were inside the zero-point estimate based on the 95% BC CI, which indicating there were no statistical difference between the specific mediating power of the two single mediation paths and the serial-multiple mediation in the ERR model. While in Table 4, the statistically significant contrast of single mediation by psychological capital and the serial-multiple mediation of perceived organizational support and psychological capital was not inside the zero-point estimate based on the 95% BC CI. Based on the contrasting pairs of specific direct effects, the path through single mediation by psychological capital was observed to have stronger mediating power than the path through serial-multiple mediation in the overcommitment model.

## Discussion

The prevalence of insomnia symptoms among nurses in this study was 57.3%, which almost the same as frontline nurses fight against COVID-19 in Wuhan, China during the early time of the pandemic (32). Worked more than 40 h a week, with chronic diseases, experienced negative life events, and worked in the emergency department was related with increased insomnia symptoms. These factors have long been recognized as risk factors for insomnia in healthcare workers (33–35). The relationship between occupational stress and insomnia has long been confirmed (11, 36). Individuals may experience a lighter sleep, increased awakenings and sleep fragmentation when sustained stress leads to the activation of HPA axis (37).

The results of the present study suggest that occupational stress has a direct negative impact on insomnia among Chinese nurses. Meanwhile, overcommitment explained insomnia better than ERR, so intrinsic stress played a more critical role than extrinsic stress in insomnia among nurses. Organization is an important source of social and emotional resources for employees. As an external resource, perceived organizational support plays an important role in mitigating or alleviating the negative effects of occupational stress and improving mental health among employees. Attention to employees' welfare and recognition of their contributions will reduce employees' occupational pressure. Several studies have confirmed that perceived organizational support was one of the protective factors for organizational behaviors and psychological outcomes in healthcare workers, and employees with supportive settings were more likely to show mental wellbeing (5, 38, 39). The finding of this study about psychological capital was consistent with our hypothesis that it mediates the relationship between occupational stress and insomnia. Psychological capital plays an important role in reducing the negative effects related to occupational stress (40, 41). As an important internal resource, it will has a positive pushing force on individuals and enables people to buffer the negative effects of work, thereby preventing the occurrence of serious mental health problems.

To the best of our knowledge, this study was the first to examine the relationships between occupational stress, perceived organizational support, psychological capital and insomnia. Our research found that perceived organizational support and psychological capital played a chain mediating role between occupational stress and insomnia. Occupational stress not only refers to physical sensation, it is also defined as a kind of psychological state (42). According to the social exchange theory (43), occupational stress may make employees' perceptions that they are not sufficiently valued by the organization, and leading to a state of psychosocial needs unfulfillment, that is, reduced perceived organizational support. Perceived organizational support and psychological capital are not static in the process of individual growth and development, as job resources, they continuously interact with job demands (occupational stress) to promote the development of job motivation based on JD-R model (44). Nurses who perceive more organizational support in the face of occupational pressure are more likely to experience high levels of psychological capital, which was consistent with previous studies (21), and the corresponding insomnia symptoms will be reduced.

The present study has some implications for hospital administrations and nursing management. Nurses insomnia symptoms should be regularly screened. These results argue for the urgent implementation of support measures to relieve their occupational stress during this special period of epidemic prevalence, such as reducing the working hours and workload of each shift, hiring new staff, and providing free and available professional psychological counseling. Creating a supportive working environment and providing online organization support services are conducive to improve the level of perceived organizational support among nurses (34). The daily online self-learning method through WeChat (a free application that provides instant messaging services in mainland China) was effective at improving psychological capital levels (45).

This study also has some limitations. First, the cross-sectional study design could not confirm the causal relationship between variables, which still needs a longitudinal study to explore. Second, this study was conducted in one hospital. The management system and shift mode of different hospitals may have an impact on the variables. Investigations should be conducted in other regions or other hospitals to confirm the results of this study in the future. Third, among many mental health outcomes, we only evaluated the insomnia symptoms of nurses. However, we believe that the relationship between variables confirmed by the results of this study also exists in anxiety, depression, and even in other occupations.

## Conclusion

The present study was the first to explore the relationship between occupational stress and insomnia symptoms among Chinese nurses using a serial-multiple mediation model, with results indicating the prevalence rate of insomnia symptoms among Chinese nurses to be 57.3%, comparatively high under the condition of normalization of the COVID-19 pandemic. The results of the present study showed that reduced occupational stress was sequentially associated with increased perceived organizational support first and then increased psychological capital, which was in turn related to reduced insomnia symptoms. Therefore, paying attention to welfare, creating supportive working environment and investing to improve psychological capital can help alleviate insomnia symptoms of nurses.

## Data Availability Statement

The supporting data can be obtained by contacting the corresponding author by email.

## Ethics Statement

The studies involving human participants were reviewed and approved by Ethics Committee of the First Affiliated Hospital of Shandong First Medical University.

## Author Contributions

JD, ZL, HL, and CN conceived, designed the research, and wrote the manuscription. JD, ZL, XZ, PS, YH, and YL performed the research and data analyses. All authors contributed to the article and approved the submitted version.

## Funding

This work was supported by the Military Medical Innovation Project (grant number 18CXZ020).

## Conflict of Interest

The authors declare that the research was conducted in the absence of any commercial or financial relationships that could be construed as a potential conflict of interest.

## Publisher's Note

All claims expressed in this article are solely those of the authors and do not necessarily represent those of their affiliated organizations, or those of the publisher, the editors and the reviewers. Any product that may be evaluated in this article, or claim that may be made by its manufacturer, is not guaranteed or endorsed by the publisher.
